# Regulation of gastric smooth muscle contraction via Ca^2+^-dependent and Ca^2+^-independent actin polymerization

This article has been retracted.

**DOI:** 10.1371/journal.pone.0209359

**Published:** 2018-12-20

**Authors:** Sunila Mahavadi, Ancy D. Nalli, Hongxia Wang, Derek M. Kendig, Molly S. Crowe, Vijay Lyall, John R. Grider, Karnam S. Murthy

**Affiliations:** Department of Physiology and Biophysics, VCU Program in Enteric Neuromuscular Sciences, Virginia Commonwealth University, Richmond, Virginia, United States of America; Institute of Biochemistry and Cell Biology, SINGAPORE

## Abstract

In gastrointestinal smooth muscle, acetylcholine induced muscle contraction is biphasic, initial peak followed by sustained contraction. Contraction is regulated by phosphorylation of 20 kDa myosin light chain (MLC) at Ser^19^, interaction of actin and myosin, and actin polymerization. The present study characterized the signaling mechanisms involved in actin polymerization during initial and sustained muscle contraction in response to muscarinic M3 receptor activation in gastric smooth muscle cells by targeting the effectors of initial (phospholipase C (PLC)-β/Ca^2+^ pathway) and sustained (RhoA/focal adhesion kinase (FAK)/Rho kinase pathway) contraction. The initial Ca^2+^ dependent contraction and actin polymerization is mediated by sequential activation of PLC-β1 via Gα_q_, IP_3_ formation, Ca^2+^ release and Ca^2+^ dependent phosphorylation of proline-rich-tyrosine kinase 2 (Pyk2) at Tyr^402^. The sustained Ca^2+^ independent contraction and actin polymerization is mediated by activation of RhoA, and phosphorylation of FAK at Tyr^397^. Both phosphorylation of Pyk2 and FAK leads to phosphorylation of paxillin at Tyr^118^ and association of phosphorylated paxillin with the GEF proteins p21-activated kinase (PAK) interacting exchange factor α, β (α and β PIX) and DOCK 180. These GEF proteins stimulate Cdc42 leading to the activation of nucleation promoting factor N-WASP (neuronal Wiskott-Aldrich syndrome protein), which interacts with actin related protein complex 2/3 (Arp2/3) to induce actin polymerization and muscle contraction. Acetylcholine induced muscle contraction is inhibited by actin polymerization inhibitors. Thus, our results suggest that a novel mechanism for the regulation of smooth muscle contraction is mediated by actin polymerization in gastrointestinal smooth muscle which is independent of MLC_20_ phosphorylation.

## Introduction

The current understanding of the molecular mechanisms that lead to smooth muscle contraction is based on the phosphorylation of the 20- kDa myosin II regulatory light chain (MLC_20_), an essential requirement for both initiating and sustaining contraction. The phosphorylation of MLC_20_ enhances the ability of actin to activate myosin-Mg^2+^-ATPase and stimulate hydrolysis of ATP on the myosin head [1–3]. The chemical energy derived from actin-activated actomyosin is converted into mechanical force that induces both cyclical sliding of overlapping actin and myosin filaments (cross-bridge cycles and cell shortening) [1–4]. Although cross-bridge cycling is essential for generating force, it does not provide a mechanism for transmitting force across the cell or between cells. It is increasingly evident that in order to transmit force, the sliding actomyosin filaments must be anchored to the opposing sides of a smooth muscle cell, as well as to other smooth muscle cells via the extra cellular matrix (ECM). This anchoring process occurs as part of a dynamic, stimulus-driven reorganization of cytoskeletal proteins at membrane adhesion junctions [5].

Upon stimulation, contraction of smooth muscle occurs in two phases: an initial Ca^2+^-dependent contraction followed by a sustained Ca^2+^-independent contraction, with minimal overlap. Initial contraction involves sequential activation of Gα_q_ and PLC-β1 by G protein-coupled receptors, resulting in inositol 1,4,5-trisphosphate (IP_3_) formation, IP_3_-dependent Ca^2+^ release via IP_3_R-1/Ca^2+^ channels, increase in cytosolic Ca^2+^ ([Ca^2+^]_*i*_), activation of Ca^2+^-calmodulin-dependent myosin light chain kinase (MLCK), and MLC_20_ phosphorylation [3,6–10].

The initial transient phase is followed by a sustained contraction. The phosphorylation of MLC_20_ during this phase is mediated by relatively weak Ca^2+^-independent MLCKs (eg, ZIP kinase) that derive their effectiveness from concurrent inhibition of MLCP and involve sequential activation of Gα_13_, the Rho-specific guanine nucleotide exchange factor (GEF), p115RhoGEF, and RhoA. RhoA activates two downstream effectors: Rho kinase (mainly Rho-associated, coiled-coil containing protein kinase 2 in smooth muscle) and phospholipase D [3]. Phospholipase D hydrolyzes phosphatidylcholine, yielding phosphatidic acid (PA) as its primary product; PA is then dephosphorylated to diacylglycerol, which activates PKC. Both Rho kinase and PKC inhibit MLCP: Rho kinase phosphorylates myosin phosphatase-targeting subunit 1 (MYPT1), the regulatory subunit of MLCP at Thr^696/855^; PKC phosphorylates the PKC potentiated inhibitor protein of 17 kDa (CPI-17), an endogenous inhibitor of MLCP, at Thr^38^, greatly enhancing its affinity for and ability to inhibit MLCP (PP1*cδ*) activity [3, 4, 11–13]. Both Rho kinase/MYPT1 and PKC/CPI-17 pathways participate in sustained muscle contraction mediated by various receptors, including M3 muscarinic receptors [9, 11–15]. Inhibitors of either Rho kinase or protein kinase C selectively block sustained contraction suggesting their specific role in mediating sustained contraction.

In addition to these pathways, well-designed studies in airway and vascular smooth muscle have highlighted the important role of cytoskeletal reorganization and actin polymerization in force transmission [2, 5, 16–18]. Instead, force transmission requires that the sliding filaments be anchored at opposite sides of smooth muscle cells. Stimulus-driven cytoskeletal reorganization involves a rapid, orderly recruitment of structural and signaling molecules to a region of the cell spanned by heterodimeric transmembrane integrin proteins. Adhesion complexes are formed upon binding of recruited molecules to the cytoplasmic region of β-integrin and/or to each other [5]. A series of interactions is initiated leading to polymerization of sub-membranous (cortical) actin into filaments that link adhesion complexes to actomyosin filaments in the cell and via integrin proteins to ECM proteins [5, 16–18].

The involvement of RhoA in focal adhesion formation and actin polymerization reflects its role as a key regulator of actin cytoskeletal organization [19, 20]. Recent studies in tracheal smooth muscle, however, appear to suggest that the main role of RhoA in the development of active tension in smooth muscle relates to its ability to regulate actin cytoskeletal dynamics, a role that may surpass that of regulating MLC_20_ phosphorylation [20]. The expression of dominant negative RhoA [T19N] abolishes actin polymerization and strongly inhibits ACh-induced contraction while having a minor effect on MLC_20_ phosphorylation, indicating that RhoA is involved in actin polymerization [21]. In contrast, the MLCK inhibitor, ML-7, strongly inhibited contraction and MLC_20_ phosphorylation but had no effect on actin polymerization [19].

The present study was designed to separately characterize the pathways that mediate actin polymerization during the initial and sustained phases of contraction in gastrointestinal smooth muscle. We postulated that during the initial phase, Ca^2+^, not RhoA, is the trigger for distinct pathways, one involving MLCK-induced MLC_20_ phosphorylation, as previously reported [1, 3, 9], the other involving Ca^2+^-dependent activation of Pyk2 (proline-rich-tyrosine kinase 2) and downstream effectors that mediate actin polymerization. Recent studies have shown that KCl-induced Ca^2+^ entry stimulates Pyk2 activity in vascular smooth muscle [22]. We assumed that IP_3_-induced Ca^2+^ release during the initial phase would activate Pyk2 and stimulate Pyk2 phosphorylation of paxillin at Tyr31 and Tyr118, the same tyrosine residues that are phosphorylated by the homologous tyrosine kinase, FAK [23]. Phosphorylation of paxillin at these sites facilitates the association of paxillin and Cdc42 GEFs, and induces sequential activation of Cdc42, N-WASP, and Arp2/3, resulting in actin polymerization. During the sustained phase, RhoA is the trigger for distinct pathways to regulate muscle contraction: one pathway involves inhibition of MLCP activity and stimulation of MLC_20_ phosphorylation via Rho kinase and PKC and the other pathway involves stimulation of actin polymerization via phosphorylation of FAK and paxillin.

## Materials and methods

### Materials

Stadie-Riggs tissue slicer was purchased from Thomas Scientific (Swedesboro, NJ); RhoA, Cdc42 and filamentous actin (F-actin) to globular actin (G-actin) (F/G-actin) ratio assay kits were purchased from Cytoskeleton (Denver, CO); the Rho kinase inhibitor Y27632 and the Arp2/3 complex inhibitor CK666 were purchased from EMD Millipore (Billerica, MA); FAK inhibitor FP 573228 and the actin polymerization inhibitors latrunculin A, and cytochalasin D were purchased from Tocris Bioscience (Bristol, UK); All PCR reagents, RNA isolation kit, TURBO DNase, SuperScript II, Lipofectamine 2000 Transfection Reagent as well as phospho-Pyk2(Tyr402) and phospho-paxillin(Tyr118) antibodies were purchased from Thermo Fisher Scientific (Rockford, IL). Anti-Arp2/3, N-WASP antibodies were purchased from Abcam (Cambridge, UK); Cdc42 antibody, phospho-FAK (pY397), and paxillin antibodies were purchased from BD Biosciences; and Cool1/β-Pix, Cool2/α-Pix, DOCK 180, and FAK antibodies were purchased from Cell Signaling Technology (Danvers, MA). Western blot supplies were purchased from Bio-Rad Laboratories (Hercules, CA). All other chemicals were purchased from Sigma-Aldrich (St. Louis, MO)

### Experimental animals

New Zealand White rabbits (weight: 4–5 lbs) were purchased from RSI Biotechnology, Clemmons, NC; and C57BL/6 mice were purchased from The Jackson Laboratories. The animals were housed in the animal facility administered by the Division of Animal Resources, Virginia Commonwealth University, and maintained in a temperature-controlled environment with free access to food and water. The rabbits were euthanized by injection of euthasol overdose (100 mg/kg); whereas mice will be anesthetized by CO_2_ inhalation/asphyxiation followed by cervical dislocation, this and all other procedures were approved by the Institutional Animal Care and Use Committee of Virginia Commonwealth University.

### Methods

#### Preparation of dispersed and cultured gastric smooth muscle cells

The rabbit antrum was separated from the rest of the stomach, and the mucosal layer was removed by sharp dissection from both fundus and antrum. Smooth muscle cells from the circular muscle layer of the stomach were isolated by sequential enzymatic digestion of muscle strips, filtration, and centrifugation as described previously [24– 27]. Antrum was cut into thin slices using a Stadie-Riggs tissue slicer and combined with fundus are incubated at 31°C for 30 min in a smooth muscle buffer (120 mM NaCl, 4 mM KCl, 2.6 mM KH_2_PO_4_, 2.0 mM CaCl_2_, 0.6 mM MgCl_2_, 25 mM HEPES, 14 mM glucose, and essential amino acid mixture 2.1% (pH7.4)) with 0.1% collagenase II (300 U/ml) and 0.01% soybean trypsin inhibitor (w/v). The partly digested tissues were washed twice with 50-ml of collagenase-free smooth muscle buffer and the muscle cells were allowed to disperse spontaneously for 30 min in collagenase-free medium. Cells were harvested by filtration through a 500 μm Nitex screen and centrifuged twice at 350 *g* for 10 min to eliminate broken cells and organelles.

Dispersed muscle cells isolated from the stomach were re-suspended in DMEM containing 200 U/ml penicillin, 200 μg/ml streptomycin, 100 μg/ml gentamycin, 2.5 μg/ml amphotericin B and 10% fetal bovine serum (DMEM-10). The muscle cells were plated at a concentration of 5× 10^5^ cells/ml and incubated at 37 °C in a CO_2_ incubator. The DMEM-10 medium was replaced every 3 days for 2–3 weeks until confluence was attained. All experiments were done on cells in the first passage [24–27].

#### Measurement of mRNA expression for FAK, paxillin, α-Pix, β-Pix and DOCK-180 by RT-PCR

Total RNA was extracted from cultured gastric smooth muscle cells by treatment with RNAqueous reagent, and contaminant genomic DNA was removed by treatment with TURBO DNase as described previously [25, 27]. RNA from each preparation was reversely transcribed using the SuperScript II system containing 50 mM Tris–HCl (pH 8.3), 75 mM KCl, 3 mM MgCl_2_, 10 mM dithiothreitol (DTT), 0.5 mM deoxynucleoside triphosphates (dNTP), 2.5 μM random hexamers and 200 units of reverse transcriptase (RT) in a 20 μl reaction volume. The reactions were carried out at room temperature for 10 min, then at 42°C for 50 min, and terminated by heating to 70°C for 15 min. Three μl of the reverse transcription complementary DNA (RT cDNA) were amplified in a final volume of 50 μl by PCR in standard conditions (2 mM MgCl_2_, 200 μM dNTP, and 2.5 units Taq polymerase) with specific primers for FAK, Cool2/PAK interacting exchange factor alpha (Cool2/αPix), Cool2/PAK interacting exchange factor beta (Cool1/βPix), paxillin, and DOCK 180. The primers were designed based on conserved sequences in human, rat, and mouse cDNAs (Table 1). PCR was performed for 30 cycles. For each experiment, a parallel control without RT was processed. The amplified PCR products were analyzed on 1.5% agarose gel containing 0.1 μg/ml ethidium bromide [25, 27].

**Table 1:** 

Primer Name	Forward 5----------3’	Reverse 5-----------3’	bp
**FAK**	**TGTGCACACTTGGAGAGCTGA**	**AGGACAATTTGGAGGCATTGGT**	**443**
**α-pix**	**ACTGCTCCACTTACCAAG**	**TTGGCAGAGTGTCTGTTGAAATGT**	**204**
**β-pix**	**CATGGCAAGGCACTGACCTGA**	**CCCATYCTGTAACTATGGGCTGT**	**166**
**DOCK 180**	**ACTCAAGAGTCCCTGCAACT**	**ATGGCCTCCTCCCACATCT**	**782**
**Paxillin**	**TCCTCTGCCACCAGGGAGCT**	**GACCAAAGAAGGCTCCACA**	**475**

#### Assay for phosphoinositide hydrolysis

Phosphoinositide hydrolysis was determined from the formation of total inositol phosphates using anion exchange chromatography as described previously [26]. Cultured smooth muscle cells were labeled with myo[^3^H] inositol (0.5 μCi) for 24 h in inositol-free DMEM. The cells were washed with PBS and treated with 1 μM acetylcholine (ACh) for 1 min in the presence and absence of 10 μM phospholipase C (PLC) -β inhibitor (U73122) for 10 min or 1 μM of actin polymerization inhibitor, latrunculin for 1 h. The reaction was terminated by adding 940 μl of chloroform/methanol/HCl (50:100:1, by volume). After extraction with 340 μl of chloroform and 340 μl of H_2_O, the aqueous phase was applied to DOWEX AG-1 columns; [^3^H]inositol phosphates were eluted, and radioactivity was determined in a liquid scintillation counter.

#### Measurement of [Ca^2+^]_i_ in muscle cells

ACh-induced increase in [Ca^2+^]_*i*_ was measured by fluorescence in a single smooth muscle cell loaded with fluorescent Ca^2+^ dye fura-2-AM. Dispersed muscle cells were plated on coverslips for 12 h in DMEM. After being washed with phosphate-buffered saline (PBS), the cells were loaded with 5 μM fura-2-AM for 1 h at room temperature. The cells were visualized through a 40× objective (0.9 numerical aperature; Carl Zeiss Microscopy, Thornwood, NY) with a Zeiss Axioskop 2 plus upright fluorescence microscope and imaged using a setup consisting of a charge-coupled device camera (Imago, TILL Photonics, Applied Scientific Instrumentation, Eugene, OR) attached to an image intensifier. The cells were alternately excited at 380 nm and 340 nm. The background and autofluorescence were corrected using images of a cell without the fura-2-AM [24].

#### Transfection of dominant-negative RhoA (RhoA [T19N]), or dominant-negative Cdc42 (Cdc42 [T17N]) in cultured gastric smooth muscle cells

Dominant-negative mutants of RhoA (RhoA [T19N]) or Cdc42 (Cdc42 [T17N]) cDNAs were subcloned into the multiple cloning site (EcoRI) of the eukaryotic expression vector pcDNA3. Recombinant plasmid DNAs (2 μg each) were transiently transfected into smooth muscle cells in primary culture using Lipofectamine 2000 Transfection Reagent for 48 h. The cells were co-transfected with 1 μg of pGreen Lantern-1 to monitor transfection efficiency. Control cells were co-transfected with 2 μg of vector (pcDNA3) and 1 μg of pGreen Lantern-1 DNA. Transfection efficiency (85% of the cells) was monitored by the expression of green fluorescent protein using FITC filters [15].

#### Determination of RhoA and Cdc42 activation

RhoA and Cdc42 activation were determined by using pull-down assays for activated RhoA or activated Cdc42, respectively. Muscle cells were solubilized in lysis buffer plus protease and phosphatase inhibitor containing 1% NP-40, 50 mM Tris-HCl, (pH 7.4), 150 mM NaCl, 10% glycerol, 2 mM EDTA, 2 mM benzamidine, 0.5 mM aprotinin, 1 mM PMSF, 2 mM sodium orthovandate, 2 mM molybdate, and 2 mM sodium pyrophosphate for 5 min at 4°C. For the analysis of RhoA activation, extracted proteins were reacted with a peptide for the glutathione S-transferase-tagged Rho-binding domain region of Rhotekin, which has a high affinity for GTP-Rho. For the analysis of Cdc42 activation, the extracted proteins were reacted with GST-PAK binding domain (PBD). Activated GTP-bound RhoA or Cdc42 were affinity-precipitated by glutathione beads and quantitated by Western blot [19].

#### Phosphorylation of paxillin, FAK, Pyk2, and MLC_20_ by western blot

Phosphorylation of FAK and Pyk2 was measured by Western blot using a phospho-specific antibody. Cultured gastric smooth muscle cells (2 × 10^6^cell/ml) were treated with 1 μM ACh and solubilized on ice for 1 h in medium containing 20 mM Tri-HCl (pH 8.0), 1 mM DTT, 100 mM NaCl, 0.5% SDS, 0.75% deoxycholate, 1 mM PMSF, 10 mg/ml leupeptin, and 100 mg/ml of aprotinin. The proteins were resolved by SDS-PAGE and electrophoretically transferred onto polyvinylidene difluoride membranes. The membranes were incubated for 12 h either with phospho-specific paxillin (Tyr118) antibody (1:1,000), phospho-specific FAK (Y397) antibody (1:1,000), phospho-specific Pyk2 (Y402) antibody (1:1,000) or phospho-specific MLC_20_ (Ser19) antibody and then for 1hr with horse-radish-peroxidase-conjugated secondary antibody (1:5,000). The protein bands were identified by enhanced chemiluminescence reagent [15, 24, 25].

#### Phosphorylation of paxillin by immunocytochemistry

Phosphorylation of paxillin was also measured by immuno cytochemistry. Rabbit gastric smooth muscle cells were cultured in an 8-well chamber slide for 2 d and treated with 1 μM ACh for 10 min in the presence or absence of 10 μM of Rho kinase inhibitor Y27632 for 10 min, or 10 μM of FAK inhibitor PF 573228 for 10 min. Cells were fixed in 4% paraformaldehyde for 20 min and incubated with blocking solution containing 5% normal donkey serum in PBS for 1 h followed by incubation with phospho-specific paxillin (Tyr118) (1:200) for 2 h at room temperature. Cells were rinsed twice in PBS and then incubated with fluorochrome-conjugated antibody for 1 h at room temperature. Cells were rinsed twice in PBS, once in water, and then mounted on glass microscope slides and analyzed under a fluorescent photomicroscope (Carl Zeiss Microscopy). Immunostaining in the absence of primary or secondary antibody was assessed for background evaluation.

#### Protein-protein association (paxillin:Cool2/α-Pix, paxillin:Cool1/β-Pix, paxillin:DOCK 180 and N-WASp:Arp2)

Associations between paxillin and cool2/α-Pix, paxillin and cool1/β-Pix, paxillin and DOCK 180 were determined by immunoprecipitation with paxillin and immunoblot with Cool2/α-Pix, Cool1/β-Pix and DOCK-180 antibodies. N-WASp and Arp2/3 associations were determined by immunoprecipitation with N-WASp and immunoblot with Arp2/3 antibody. Cultured gastric smooth muscle cells (2 × 10^6^cell/ml) were treated with 1 μM ACh for 5 min and then solubilized on ice for 1 h in medium containing 20 mM Tris-HCl (pH 8.0), 1 mM DTT, 100 mM NaCl, 0.5% SDS, 0.75% deoxycholate, 1 mM PMSF, 10 mg/mL of leupeptin, and 100 mg/mL aprotinin. The immunoprecipitated proteins were resolved by SDS-PAGE, and electrophoretically transferred onto polyvinylidene difluoride membranes. The membranes were incubated for 12 h with primary antibody (1:1,000), and then for 1h with horse-radish-peroxidase-conjugated secondary antibody (1:5,000). The protein bands were identified by enhanced chemiluminescence reagent [25].

#### In situ proximity ligation assay (PLA)

Duolink *in situ* proximity ligation assays (PLA) were performed to detect cellular interactions between paxillin and PIX or paxillin and DOCK 180. PLA yields a fluorescent signal when the target proteins are localized within 40 nm of each other. Cultured rabbit gastric smooth muscle cells were treated with 1 μM of ACh or left untreated and then fixed, permeabilized and incubated with primary antibodies followed by secondary antibodies conjugated to PLA probes. Duolink hybridization, ligation, amplification, and detection media were administered according to the manufacturer’s instructions. Randomly selected cells from both untreated and ACh treated groups were analyzed for paxillin-α PIX, paxillin-β PIX and paxillin-DOCK 180 interactions by visualizing Duolink fluorescent spots using a Zeiss fluorescence microscope in a single Z-line scan through the middle of the cell.

#### Analysis of F-actin and G-actin

Actin polymerization is characterized by an increase in F/G-actin ratio [19, 20, 28]. The relative proportions of F-actin and G-actin in cultured gastric smooth muscle cells were analyzed using an F/G-actin assay kit. Cultured gastric smooth muscle cells were homogenized in 200 μl of F-actin stabilization buffer containing 50 mM PIPES (pH 6.9), 50 mM NaCl, 5 mM MgCl_2_, 5 mM EGTA, 5% glycerol, 0.1% Triton X-100, 0.1% Nonidet P-40, 0.1% Tween 20, 0.1% β-mercaptoethanol, 0.001% antifoam, 1 mM ATP, 1 μg/ml pepstatin, 1 μg/ml leupeptin, 10 μg/ml benzamidine, and 500 μg/ml tosyl arginine methyl ester. Supernatants of the protein extracts were collected after centrifugation (150,000 *g* for 60 min at 37°C). The pellets were resuspended in 200 μl of F-actin depolymerization buffer containing 10 μM cytochalasin D and then incubated on ice for 1 h to depolymerize F-actin. The resuspended pellets were gently mixed every 15 min. Ten microliters of supernatant (G-actin) and pellet (F-actin) fractions were subjected to immunoblot analysis using anti-actin antibody. The relative amounts of F-actin and G-actin were determined using densitometry [19]. The cumulative data were normalized to the basal ratio to 1.

#### Insertion of RhoA (RhoA [T19N]) and RhoA [His]6 plasmids into gastric smooth muscle strips

Dominant-negative RhoA (RhoA [T19N]) and RhoA [His]6 plasmids were introduced into gastric smooth muscle strips by reversible permeabilization method. Immediately after the optimal smooth muscle length was determined, the muscle strips were put onto metal hooks with tension in order to keep the strips at a certain length. These strips were incubated in each solution listed: solution 1 containing (in mM) 10 EGTA, 5 Na_2_ATP, 120 KCl, 2 MgCl_2_, and 20 N-tris (hydroxymethyl)methyl-2-aminoethanesulfonic acid (TES) at 4°C for 120 min; solution 2 containing (in mM) 0.1 EGTA, 5 Na_2_ATP, 120 KCl, 2 MgCl_2_, and 20 TES, as well as 20 μg/ml plasmids (pCDNA3 RhoA(His)6 or pCDNA3 RhoA[T19N]) at 4°C for overnight; solution 3 containing (in mM) 0.1 EGTA, 5 Na_2_ATP, 120 KCl, 10 MgCl_2_, and 20 TES at 4°C for 30 min; and solution 4 containing (in mM) 110 NaCl, 3.4 KCl, 0.8 MgSO_4_, 25.8 NaHCO_3_, 1.2 KH_2_PO_4_, and 5.6 dextrose at 22°C for 60 min. Solutions 1–3 were aerated with 100% O_2_ to maintain pH 7.1, and solution 4 was aerated with 95% O_2_-5% CO_2_ to maintain pH 7.4. CaCl_2_ was added to solution 4 after 30 min gradually in order to achieve a final concentration of 2.4 mM. After insertion of the plasmids into the muscle strips, the muscle strips were then transferred to DMEM containing 5 mM Na_2_ATP, 100 U/ml penicillin, 100 μg/ml streptomycin, 50 μg/ml kanamycin and 20 μg/ml plasmids (pCDNA3 vector or pCDNA3 RhoA (His)6 or pCDNA3 RhoA[T19N] and incubated at 37°C for 2 days to allow for expression of the recombinant proteins. After 2 days muscle strips were transferred into Krebs buffer containing (in mM) 118 NaCl, 4.75 KCl, 1.19 KH_2_PO_4_, 1.2 MgSO_4_, 2.54 CaCl_2_, 25 NaHCO_3_, 11 mM glucose (pH 7.4) at 37°C in 5 or 2 ml baths and attached to force transducers for the immediate measurement of isometric force.

After measurement of isometric force, the muscle cells were isolated from muscle strips, (*see method described in Preparation of dispersed and cultured gastric smooth muscle cells*) cells were poured over glass coverslips, and allowed to adhere to the coverslips for 3–4 h at 37°C 10% CO_2_ incubator in a humidity chamber. Cells were fixed for 20 min in 4% paraformaldehyde (vol/vol) in phosphate-buffered saline (PBS) (in mM: 137 NaCl, 4.3 Na_2_HPO_4_, 1.4 KH_2_PO_4_, and 2.7 KCl, pH 7.4) and incubated with blocking solution containing 5% normal donkey serum in PBS for 1 h followed by overnight incubation with (His)6 antibody at 4°C. Cells were rinsed twice in PBS and then incubated with fluorochrome-conjugated antibody for 1 h at room temperature. Cells were rinsed twice in PBS, once in water, and then mounted on glass microscope slides and analyzed under a fluorescent photomicroscope (Carl Zeiss Microscopy).

#### Measurement of smooth muscle contraction by organ bath

Muscle strips from the fundus or antrum of the stomach from mice were collected and rinsed with PBS. The muscle strip was tied at each end with silk thread and mounted vertically in 5 ml tissue bath containing oxygenated (95% O_2_/5%CO_2_) Kreb’s solution at a pH of 7.4 at 37 °C containing 118 mM NaCl, 4.8 mM KCl, 1mM MgSO_4_, 1.15 mM NaH_2_PO_4_, 15 mM NaHCO_3_, 10.5 mM glucose and 2.5 mM CaCl_2_. The tissues were mounted between glass rod and isometric transducers (Grass Technologies) connected to a computer recording system (Polyview). Preparations were allowed to equilibrate for 1h at resting tension (1g) before initiation of experiments and bath buffer solution was changed every 15 minutes during equilibration. To measure the contraction, strips were treated with 10 μM acetylcholine (ACh). Contraction was measured in the absence of TTx. In addition, control muscle strips were treated with ACh in the presence or absence of IP_3_ receptor inhibitor (Xestospongin C, 10 μM; 15 min), Ca^2+^ chelator (BAPTA, 10 μM; 15 min), MLCK inhibitor (ML-9, 10 μM; 15 min), Rho kinase inhibitor (Y27632, 10 μM; 15 min), FAK inhibitor (PF573228, 10 μM; 15 min), Arp2/3 inhibitor (CK666, 200 μM; 1h), and actin polymerization inhibitors (cytochalasin D, 10 μM; 1h and latrunculin, 1 μM; 1h). At the end of each experiment, the strips were blotted dry and weighed (tissue wet weight). Muscle strips from mouse stomach consisting of either fundus alone or fundus with small amounts of antrum were used. However, most of the tracings are from the responses from fundus. Any phasic activity reflects responses from strips containing antral tissue. In all strips, only the peak initial peak and sustained contractions were measured.

#### Measurement of smooth muscle contraction by scanning micrometry

Muscle cell contraction was measured in freshly dispersed muscle cells by scanning microscopy as described previously (24–26). Cell aliquots containing 10^4^ muscle cells/ml were treated with 1 μM ACh for 30 s and 5 min in the presence or absence of 10 μM MLCK inhibitor ML-9 for 10 min, 2 μg/ml of RhoA inhibitor C3 exoenzyme for 2 h, 10 μM of Rho kinase inhibitor Y27632 for 10 min, 10 μM of FAK inhibitor PF573228 for 1 h, 1 and 10 μM of the actin polymerization inhibitors latrunculin, an agent derived from sponges, which binds to monomeric actin (G-actin) and prevents its polymerization, and cytochalasin D, an agent derived from fungi, which binds to barbed end of (+ end) F-actin to block further subunit addition for 1 h and 200 μM of Arp2/3 complex for 1 h; the reaction was terminated with 1% acrolein. The lengths of muscle cells treated with ACh alone and in the presence of various inhibitors were compared with the lengths of untreated cells, and contraction was expressed as the percentage of decrease in cell length compared with control.

#### Statistical analysis

The results were expressed as means ± SE of *n* experiments and analyzed for statistical significance by Student's *t*-test for paired and unpaired values. Differences among groups were tested by ANOVA and checked for significance via Fisher's protected least significant difference test. *P* < 0.05 was considered significant.

## Results

### Expression of FAK, paxillin, α-Pix, β-Pix and DOCK 180 in gastric smooth muscle cells

FAK, paxillin, α-Pix, β-Pix and DOCK 180 were detected by RT-PCR and western blot in cultured rabbit gastric smooth muscle cells and in brain homogenates. The PCR products of expected size were obtained with specific primers for FAK (443 bp), paxillin (475 bp), Cool2/α-PIX (204 bp), Cool1/β-PIX (166 bp), DOCK 180 (782 bp) (Fig 1*A*); expected protein size was obtained with specific antibodies for FAK (125 kDa), paxillin (68 kDa), α-PIX (87 kDa), β-PIX (81 kDa), DOCK 180 (215 kDa) (Fig 1*B*).

**Fig 1:** Expression of focal adhesion kinase (FAK), paxillin, Cool2/p21-activated kinase (PAK) interacting exchange factor alpha (Cool2/α-Pix), Cool1/ p21-activated kinase (PAK) interacting exchange factor beta (Cool1/β-Pix) and DOCK 180 in smooth muscle cells. *A*: Total RNA was isolated from cultured gastric smooth muscle cells and brain homogenates as control were reverse transcribed (RT). PCR products of expected-size FAK (443 bp), paxillin (475 bp), Cool2/α-Pix (204 bp), Cool1/β-Pix (166 bp), and DOCK 180 (782 bp) were obtained in muscle cells and in brain homogenates. B: Western blot analysis showed that corresponding proteins with appropriate molecular weights were obtained in muscle cells and in brain homogenates (40 μg protein). MW, molecular weight.

### Increase of paxillin phosphorylation via RhoA-mediated FAK by ACh

Activation and recruitment of FAK by RhoA phosphorylates adaptor protein paxillin, which is crucial for actin polymerization [19]. Treatment of cultured gastric smooth muscle cells with 1 μM ACh for 10 min significantly increased RhoA activation by 110%±12%. However, this increase in RhoA activation was abolished in cells expressing RhoA dominant negative (RhoA [T19N]) (Fig 2*A*). Treatment of cultured gastric smooth muscle cells with 1 μM ACh for multiple time periods resulted in a significant increase in FAK phosphorylation at Tyr397. For example, the phosphorylation of FAK was 350% ± 40% increase at 5 min (Fig 2*B*). Consistent with the increase in activation of RhoA and FAK, treatment of cultured gastric smooth muscle cells with 1 μM ACh for 10 min significantly increased the phosphorylation of paxillin at Tyr118 by 125% ± 15%. The increase in phosphorylation of paxillin was significantly inhibited in cells expressing RhoA dominant negative (RhoA [T19N]) (by 88% ± 10% decrease) (Fig 3*A*). Treatment of cultured gastric smooth muscle cells with FAK inhibitor PF573228 abolished ACh-induced increase in paxillin phosphorylation (Fig 3*B* and 3*C*). Treatment of smooth muscle cells with Rho kinase inhibitor Y27632 had no effect on paxillin phosphorylation in response to ACh (125% ± 15% vs 120% ± 10% increase) (Fig 3*B* and 3*C*).

**Fig 2:** Stimulation of RhoA activity and phosphorylation of FAK by acetylcholine (ACh). *A*: Cultured smooth muscle cells expressing either control vector or RhoA dominant negative (RhoA [T19N]) were treated for 10 min with 1 μM ACh. Immunoprecipitates derived from 500 μg of protein using the glutathione S-transferase-tagged Rho-binding domain region of Rhotekin beads were separated using SDS-PAGE and immunoblotted using RhoA antibody; the results are expressed as densitometric values. Values are means ± SE of four experiments. *B*: Immunoblots of FAK and phospho-FAK (Y397) from extracts of smooth muscle cells either unstimulated or stimulated with 1 μM ACh for different time periods ≤ 5 min. Phosphorylation of FAK was measured using phospho-specific Tyr FAK (Y397) antibody. The results are expressed as densitometric values. Values are means ± SE of five experiments. **P<0.001, ## *P*<0.01.

**Fig 3:** Stimulation of paxillin phosphorylation by ACh. *A*: Cultured smooth muscle cells expressing either control vector or RhoA dominant negative (RhoA [T19N]) were treated for 10 min with 1 μM ACh. Phosphorylation of paxillin was measured using phospho specific Tyr paxillin antibody (Y118) and results are expressed as densitometric values. Values are means ± SE for three experiments. *B*: Immunostaining of paxillin phosphorylation in cultured smooth muscle cells were treated with 1 μM ACh for 10 min in the presence or absence of Rho kinase inhibitor Y27632 (10 μM, 10 min), FAK inhibitor PF 573228 (10 μM, 10 min). *C*: Immunoblots of paxillin and phospho paxillin from extracts of smooth muscle cells either unstimulated or stimulated with 1 μM ACh in the presence or absence of Rho kinase inhibitor Y27632 (10 μM, 10 min), or FAK inhibitor PF 573228 (10 μM, 10 min). Phosphorylation of paxillin was measured using phospho-specific Tyr118 paxillin antibody. The results are expressed as densitometric values. Values are means ± SE of four experiments. **P<0.001.

### Increase of paxillin association with GEFs via RhoA by ACh

Phosphorylation of paxillin facilitates the ability of adaptor proteins to bind to DOCK 180 and α/β PIX [19, 20]. Consistent with the increase in phosphorylation of paxillin, treatment of the cultured gastric smooth muscle cells with 1 μM ACh for 10 min significantly increased the number of fluorescent spots, indicating many interactions between paxillin- Cool2/α-PIX (Fig 4*A*), paxillin- Cool1/β-PIX (Fig 4*B*) and paxillin-DOCK180 (Fig 4*C*) measured by Duolink *in situ* PLA. Also, the association of paxillin with Cool2/α-PIX (by 180% ± 20% increase) (Fig 4*D*), Cool1/β-PIX (by 148% ± 16% increase) (Fig 4*E*) and DOCK 180 (by 120% ± 12% increase) (Fig 4*F*) measured by immunoprecipitation and immunoblot were increased by ACh. However, the increased association of Cool2/α-PIX (89% ± 10% decrease) (Fig 4*D*) and Cool1/β- PIX (86% ± 8% decrease) (Fig 4*E*) was significantly inhibited in cells expressing RhoA dominant negative (RhoA [T19N]), whereas, DOCK 180 was abolished in cells expressing RhoA dominant negative (RhoA [T19N]) (Fig 4*F*).

**Fig 4:** Protein-protein association. Cultured smooth muscle cells expressing either control vector or RhoA dominant negative (RhoA [T19N]) were treated for 10 min with 1 μM ACh. The association of paxillin with α-Pix (*A and D*), paxillin with β-Pix (*B and E*), and paxillin with DOCK 180 (*C and F*) are shown. Immunoprecipitates derived from 100 μg protein using paxillin antibody were separated using SDS-PAGE and immunoblotted using α-Pix, β-Pix and DOCK 180 antibodies. The results are expressed as densitometric values. Values are means ± SE of three experiments. **P<0.001.

### Increased Cdc42 activation via RhoA by ACh

Consistent with the increased association of paxillin with cool2/α-PIX, cool1/β-PIX and DOCK-180 GEF proteins, we found that treatment of cultured gastric smooth muscle cells with 1 μM of ACh for 10 min significantly increased Cdc42 activation (by 80% ± 8%) (Fig 5*A*). The increase in Cdc42 activation was abolished in cells expressing RhoA dominant negative (RhoA [T19N]) (Fig 5*A*).

**Fig 5:** Activation of Cdc42 and N-WASP:Arp-2/3 complex association. *A*: Cultured smooth muscle cells expressing either control vector or RhoA dominant negative (RhoA [T19N]) were treated for 10 min with 1 μM ACh. Immunoprecipitates derived from 500 μg of protein using glutathione S-transferase-tagged p21-activated kinase (PAK) binding domain (PBD) beads were separated using SDS-PAGE and immunoblotted using Cdc42 antibody, and the results are expressed as densitometric values. Values are means ± SE for four experiments. *B*: Cultured smooth muscle cells expressing control vector or RhoA dominant negative (RhoA [T19N]) or Cdc42 dominant negative (Cdc42 [T17N]) were treated for 10 min with 1 μM ACh. Immunoprecipitates derived from 100 μg of protein using the N-WASP antibody were separated using SDS-PAGE and immunoblotted using Arp2/3 antibody. The results are expressed as densitometric values. Values are means ± SE of four experiments. **P<0.001.

### Increase in N-WASP association with Arp2/3 by ACh

Activation of N-WASP, which is an actin regulatory protein, is directly regulated by the small GTPase Cdc42 [29–32]. Rac or RhoA GTPases cannot bind directly to WASP family proteins; thus, RhoA cannot directly regulate N-WASP activity [33, 34]. The activation of N-WASP causes its association with Arp2/3 to initiate actin polymerization [35]. Consistent with the increase in activation of Cdc42, treatment of cultured gastric smooth muscle cells with 1 μM ACh for 10 min significantly increased the association of N-WASP with Arp2/3 (125% ± 13% increase) (Fig 5*B*). However, the increase in association of N-WASP with Arp2/3 was abolished in cells expressing RhoA dominant negative (RhoA[T19] and in cells expressing Cdc42 dominant negative (Cdc42 [T17N]) (Fig 5*B*).

### Increased sustained F/G-actin ratio via RhoA/FAK/Cdc42 by ACh

Consistent with the increase in the activation of Cdc42 and the association of N-WASP with Arp2, treatment of gastric smooth muscle cells with 1 μM ACh for 10 min significantly increased the F/G-actin ratio, reflecting an increase in actin polymerization (90% ± 10% increase) (Fig 6*A*). This increase in actin polymerization was abolished in cells expressing RhoA dominant negative (RhoA [T19N] (Fig 6*A*) and by 10 μM of FAK inhibitor PF573228 *(*Fig 6*B*). However, there was no significant effect on actin polymerization by the Rho kinase inhibitor Y27632 (91% ± 10% increase vs 89% ± 8% increase) (Fig 6*B*). Also, the increase in actin polymerization by ACh was significantly inhibited in cells expressing dominant-negative Cdc42 (Cdc42 [T17N]) (91% ± 10% increase vs 15% ± 2% increase) (Fig 6*C*), by 200 μM of the Arp 2/3 complex inhibitor CK666 (91% ± 10% increase vs 1% ± 0.2% increase) (Fig 7*A*). Treatment of gastric culture smooth muscle cells with 1 μM latrunculin or 10 μM cytochalasin D abolished ACh-induced F/G-actin ratio (Fig 7*B*).

**Fig 6:** RhoA/FAK/Cdc42-mediated increase in sustained actin polymerization by ACh. *A*: Actin polymerization (F/G-actin) was measured by western blot using actin antibody. Cultured smooth muscle cells expressing either control vector or RhoA dominant negative (RhoA [T19N]) were treated for 10 min with 1 μM ACh. *B*: Cultured smooth muscle cells were pre- treated with the Rho kinase inhibitor Y27632 (10 μM, 10 min) or the FAK inhibitor PF573228 (10 μM, 1 h) followed by 1 μM ACh for 10 min. *C*: Cultured smooth muscle cells expressing either control vector or Cdc42 dominant negative Cdc42 [T17N] were treated for 10 min with 1 μM ACh. The results are expressed as densitometric values. Values are means ± SE of five to six experiments. **P<0.001.

**Fig 7:** Arp2/3 complex-mediated increase in sustained actin polymerization by ACh. Cultured smooth muscle cells were pre-treated with Arp2/3 inhibitor (CK-666, 200 nM) *A*: or actin polymerization inhibitors (cytochalasin D, latrunculin, 10 μM) *B*: followed by 1 μM ACh for 10 min. Actin polymerization (F/G-actin) was measured by western blot using actin antibody. The results are expressed as densitometric values. Values are means ± SE of three experiments. **P<0.001.

### Increased of sustained muscle contraction via RhoA-mediated Rho kinase, FAK and initial muscle contraction via MLCK and actin polymerization by ACh

Treatment of dispersed smooth muscle cells with 1 μM ACh for 10 min significantly increased sustained muscle contraction. This increase was significantly inhibited by a variety of substances: C3 exoenzyme (81% ± 9% decrease), Rho kinase inhibitor alone (71% ± 7% decrease), FAK inhibitor alone (69% ± 8% decrease), a combination of Rho kinase inhibitor and FAK inhibitor (93% ± 10% decrease), the actin polymerization inhibitors cytochalasin D (78% ± 8% decrease), latrunculin (80% ± 8% decrease), and Arp 2/3 inhibitor CK666 (76% ± 7% decrease), though not by the MLCK inhibitor ML-9. (Fig 8a). Treatment of gastric smooth muscle cells with 1 μM ACh for 1 min significantly increased MLC_20_ phosphorylation and initial muscle contraction. The increase in MLC_20_ phosphorylation was inhibited by ML-9, but was not affected with actin polymerization inhibitor cytochalasin D (Fig 8b insert). Also, the increase in initial muscle contraction was significantly inhibited by MLCK inhibitor ML-9 (82% ± 8% decrease), Arp 2/3 complex inhibitor CK666 (80% ± 9% decrease) and actin polymerization inhibitors cytochalasin D (73% ± 7% decrease) and latrunculin (71% ± 8% decrease) (Fig 8b). Organ bath studies on mouse gastric smooth muscle strips showed that, ACh-induced sustained muscle contraction was inhibited in dominant negative mutant of RhoA (RhoA[T19N]) which was inserted in muscle strips by reversible permeabilization method (78 ± 8% decrease) (Fig 9). ACh-induced sustained muscle contraction was inhibited by Rho kinase inhibitor (65 ± 8% decrease), FAK inhibitor (72 ± 9% decrease), the actin polymerization inhibitors cytochalasin D (85 ± 9% decrease), latrunculin (82 ± 8% decrease), and Arp 2/3 inhibitor CK666 (80 ± 9% decrease) (Fig 10). Also ACh-induced initial muscle contraction was inhibited by MLCK inhibitor ML-9 (90 ± 10% decrease), Ca^2+^ chelator BAPTA (95 ± 10% decrease), IP_3_ receptor inhibitor Xestospongin C (90 ± 10% decrease), actin polymerization inhibitors cytochalasin D (80 ± 8% decrease), latrunculin ((75 ± 8% decrease), and Arp 2/3 complex inhibitor CK666 (78% ± 9% decrease) (Fig 11).

**Fig 8:** Inhibition of sustained and initial actin polymerization prevents ACh-induced sustained and initial smooth muscle contraction in muscle cells. Muscle contraction was measured by scanning micrometry. *A*: Pre-treatment of dispersed smooth muscle cells with the MLCK inhibitor ML-9 (10 μM, 10 min), RhoA inhibitor *Clostridium botulinum* C3 exoenzyme (2μg/ml, 1 h), Rho kinase inhibitor Y27632 (10 μM, 10 min), FAK inhibitor PF573228 (10 μM, 1 h) or Arp2/3 inhibitor CK-666 (200 μM, 1h), actin polymerization inhibitors (cytochalasin D, 10 μM; latrunculin, 1 μM, 1 h) was followed by 1 μM ACh for 10 min. *B*: Pre-treatment of dispersed smooth muscle cells with MLCK inhibitor, ML-9 (10 μM, 10 min), or Arp2/3 complex inhibitor, CK-666 (200 μM, 1h), and actin polymerization inhibitors (cytochalasin D, 10 μM; latrunculin, 1 μM, 1h) followed by 1 μM ACh for 1 min. The results are expressed as percentage decrease in cell length. Insert: MLC_20_ phosphorylation was measured by western blot using phospho specific antibody. Pre-treatment of cultured smooth muscle cells with MLCK inhibitor, ML-9 (10 μM, 10 min) and actin polymerization inhibitor (cytochalasin D, 10 μM, 1h) followed by 1 μM ACh for 1 min. Values are means ± SE of three experiments. **P<0.001.

**Fig 9:** Inhibition of RhoA prevents ACh-induced sustained smooth muscle contraction in muscle strips. Muscle contraction was measured as increase in sustained contraction in response to acetylcholine (10 μM) in organ bath experiments in gastric smooth muscle of mice in the presence or absence of RhoA [His]6 or dominant-negative RhoA ([T19N]). Results are expressed as mN/100 mg of tissue. Traces and immunostaining of (His)6 are included in the graph. Values are means ± SE of 4–6 experiments. **P<0.001.

**Fig 10:** Inhibition of sustained actin polymerization prevents ACh-induced sustained smooth muscle contraction in muscle strips. Muscle contraction was measured as increase in sustained contraction in response to acetylcholine (10 μM) in organ bath experiments in gastric smooth muscle of mice in the presence or absence of Rho kinase inhibitor Y27632 (10 μM, 10 min), FAK inhibitor PF573228 (10 μM, 1 h) or Arp2/3 inhibitor CK-666 (200 μM, 1h), actin polymerization inhibitors (cytochalasin D, 10 μM; latrunculin, 1 μM, 1 h). Results are expressed as mN/100 mg of tissue. Traces are included in the graph. Values are means ± SE of 4–6 experiments. **P<0.001.

**Fig 11:** Inhibition of initial actin polymerization prevents ACh-induced initial smooth muscle contraction. Muscle contraction was measured as increase in initial contraction in response to acetylcholine (10 μM) in organ bath experiments in gastric smooth muscle of mice in the presence or absence of MLCK inhibitor ML-9 (10 μM, 10 min), Ca^2+^ Chelator BAPTA (10 μM, 15 min), IP_3_ receptor inhibitor Xestospongin C (10 μM, 15 min) or Arp2/3 inhibitor CK-666 (200 μM, 1h), actin polymerization inhibitors (cytochalasin D, 10 μM; latrunculin, 1 μM, 1 h). Results are expressed as mN/100 mg of tissue. Values are means ±SE of 4–6 experiments. **P<0.001.

### Increased of initial F/G-actin ratio via PLC-β1/Ca^2+^ by ACh

Treatment of gastric smooth muscle cells with 1 μM ACh for 1 min significantly increased initial actin polymerization (by 90% ± 10%). This increase was abolished by phospholipase C-β inhibitor U73122 and calcium chelator (Fig 12*A*). However, there was no effect using the MLCK inhibitor ML-9 (90% ± 10% increase vs 95% ± 10% increase) (Fig 12*B*). In addition, ACh-induced initial actin polymerization was abolished by the actin polymerization inhibitors latrunculin A and cytochalasin D (Fig 12*C*).

**Fig 12:** Increase in initial actin polymerization by ACh. The initial actin polymerization (F-actin to G-actin) was measured by Western blot using actin antibody in the pre-treatment of cultured smooth muscle cells with PLC inhibitor U73122 (10 μM, 10 min) and, Ca^2+^ Chelator BAPTA (1 μM, 10 min) (*A*); and the MLCK inhibitor ML-9 (1 μM, 10 min) (*B*); and actin polymerization inhibitors (cytochalasin D, 10 μM; latrunculin, 1 μM 1 h) (*C*), followed by 1 μM ACh for 1 min. The results are expressed as densitometric values. Values are means ± SE of seven experiments. **P<0.001.

### Lack of effect on ACh-induced phosphoinositide (PI) hydrolysis and [Ca^2+^]_i_ by actin polymerization inhibitor latrunculin

Treatment of gastric smooth muscle cells with 1 μM ACh for 1 min significantly increased PI hydrolysis. Relative to the basal value, ACh increased PI hydrolysis by 150% ± 15% (Fig 13*A*). The ACh-induced increase in PI hydrolysis was significantly inhibited by the phospholipase C-β inhibitor U73122 (60% ± 5% decrease), but the actin polymerization inhibitor latrunculin had no effect (150% ± 15% increase vs 155% ± 18% on PI hydrolysis (Fig 13*A*). In parallel experiments ACh also increased [Ca^2+^]*i* (Fig 13*B*). Latrunculin also did not inhibit the ACh-induced increase in [Ca^2+^]_*i*_.

**Fig 13:** Lack of effect on phosphoinositide (PI) hydrolysis and [Ca^2+^]_*i*_ by actin polymerization inhibitors. *A*: PI hydrolysis in response to ACh was measured in muscle cells labeled with myo [^3^H] inositol. Cultured smooth muscle cells were pretreated with the PLC-β inhibitor U73122 (10 μM for 10 min) or, the actin polymerization inhibitor latrunculin (1 μM, 1 h) followed by 1 μM ACh for 1 min, and PI hydrolysis was measured as an increase in water-soluble [^3^H] inositol formation. PI hydrolysis is expressed as [^3^H] inositol phosphate formation in counts per minute (cpm) per mg protein. *B*: Isolated smooth muscle cells were loaded with 5 μM fura-2 and treated with 1 μM ACh in the presence or absence of the actin polymerization inhibitor latrunculin (1 μM, 1 h). The cells were alternately excited at 380 nm and 340 nm. Results are expressed as a 340/380 ratio, and an increase in ratio reflects an increase in cytosolic Ca^2+^. Values are means ± SE of ten cells. **P<0.001.

### Increased Pyk2(Y402) phosphorylation by ACh

Recent studies have shown that KCl-induced Ca^2+^ entry in smooth muscle stimulates Pyk2 activity [22]. We hypothesized that IP_3_-induced Ca^2+^ release during the initial phase would activate Pyk2. Consistent with the increase in PI hydrolysis and [Ca^2+^]_*i*_, treatment of gastric smooth muscle cells with 1 μM ACh significantly increased Pyk2 (Y402) phosphorylation in multiple time periods, with the maximum phosphorylation at 5 min (Fig 14*A*). The increase in ACh-induced Pyk2 phosphorylation (245% ± 28%) was significantly inhibited by Ca^2+^ chelator (BAPTA) (78% ± 7% decrease) (Fig 14*B*).

### Increased paxillin phosphorylation via Ca^2+^ by ACh

Experiments using aorta from Deoxycorticosterone acetate (DOCA)-salt mice indicated that the activation of paxillin is a Pyk2 target [36]. We hypothesized that the activation of Pyk2 stimulates phosphorylation of paxillin at Tyr118, the same Tyr residues phosphorylated by the homologous tyrosine kinase, FAK (23). Treatment of gastric smooth muscle cells with 1 μM ACh for 1 min significantly increased the phosphorylation of paxillin (130% ± 15%), an increase that was significantly inhibited by the Ca^2+^ chelator BAPTA (63% ± 5%) (Fig 15).

**Fig 14:** Increase in Pyk2 phosphorylation by ACh. *A*: Immunoblots of Pyk2 and phospho-Pyk2 from extracts of smooth muscle cells either unstimulated or stimulated with 1 μM ACh for different time periods ≤ 5 min. Values are means ± SE of six experiments. *B*: Immunoblots of Pyk2 and phospho Pyk2 from extracts of smooth muscle cells either unstimulated or stimulated with 1 μM ACh in the presence or absence of Ca^2+^ chelator BAPTA (10 μM, 10 min). Phosphorylation of Pyk2 was measured using phospho-specific Tyr Pyk2 (Y402) antibody. The results are expressed as densitometric values. Values are means ± SE of three experiments. **P<0.001.

**Fig 15:** Ca^2+^ mediated paxillin phosphorylation by ACh. Immunoblots of paxillin and phospho paxillin from extracts of smooth muscle cells either unstimulated or stimulated with 1 μM ACh for 1 min in the presence or absence of Ca^2+^ chelator BAPTA (10 μM, 10 min). Phosphorylation of paxillin was measured using phospho-specific Tyr paxillin (Y118) antibody. The results are expressed as densitometric values. Values are means ± SE of three experiments. **P<0.001.

## Discussion

Others and we have demonstrated that the contraction of gastrointestinal smooth muscle is mediated via the phosphorylation of MLC_20_ [1, 3, 4]. The phosphorylation levels of MLC_20_ are regulated by two enzymes: MLCK and MLCP. MLCK is a Ca^2+^/CaM-dependent enzyme. In gastrointestinal smooth muscle, activation of the muscarinic M3 receptor by ACh increases PLC-β1 activity, IP_3_ formation, Ca^2+^ release, Ca^2+^/CaM-dependent MLCK activity, and phosphorylation of MLC_20_ at Ser^19^ to cause initial muscle contraction. Sustained muscle contraction is a Ca^2+^ independent mechanism mediated by two RhoA-dependent pathways. One pathway involves the activation of RhoA, which phosphorylates MYPT1 at Thr^696^ by Rho kinase, and another pathway involves phosphorylation of CPI-17 at Thr^38^ by PKC. The phosphorylation of both MYPT1 and CPI-17 leads to the inhibition of MLCP’s catalytic activity to augment MLC_20_ phosphorylation and cause sustained muscle contraction [1, 3, 4, 11].

Actin polymerization plays a critical role in the regulation of active tension development in airway smooth muscle and a number of other smooth muscle tissues [5, 19]. Studies from multiple groups have shown that RhoA GTPase plays an important role in both the mechano-transduction pathway and agonist-induced changes in actin polymerization, but there are three different types of downstream pathways that have been suggested [37–39]. One RhoA-mediated pathway involves the formin homology domain protein 1 (FHOD1). FHOD1 is a member of the Dia1formin family. Upon activation of RhoA, FHOD1 binds to the plus-end of actin filaments and recruits actin monomers by binding to profilin [40, 41]. In the second pathway, RhoA initiates phosphorylation and subsequent inactivation of the ADF/cofilin family of actin-filament serving/depolymerizing proteins through the activation of LIM kinases. Phosphorylation of cofilin by the LIM kinase inhibits its ability to depolymerize actin filaments [38, 42]. A third pathway involves Cdc42, another small GTPase activated by RhoA through an ERK and PAK1/p38 pathway, which has been found to activate N-WASP. Phosphorylation activated N-WASp regulates actin ranching at focal adhesions in airway-differentiated smooth muscle cells and cultures of aortic smooth muscle cells [43, 44].

In the present study, we provide a novel mechanism of the signaling pathways that mediate a Ca^2+^ dependent and independent contraction via actin polymerization in gastrointestinal smooth muscle. The signaling molecules, such as FAK, paxillin, α-Pix, β-Pix, and DOCK-180 proteins, are involved in actin polymerization and are expressed in gastric smooth muscle cells. Treatment of muscle cells with ACh induced muscle contraction is biphasic, with an initial Ca^2+^ dependent phase that occurs via initial actin polymerization and a sustained Ca^2+^ independent phase that occurs via sustained actin polymerization. In most cell types, actin cytoskeletal dynamics and organization are mediated by RhoA [37–39]. Our results replicate that treatment of muscle cells with ACh induced RhoA activation and FAK activation, which is involved in the actin polymerization.

Activation and recruitment of FAK by RhoA from the cytosol to focal adhesions is a critical early step in the process that leads to actin polymerization. FAK consists of an N-terminal FERM (protein 4.1, ezrin, radixin, and moesin homology) domain, a central kinase domain, proline-rich regions, and a C-terminal focal adhesion-targeting (FAT) domain [23]. Auto-phosphorylation of FAK at Tyr397 creates a motif recognized by src-homology-2 (SH2)-containing proteins such as Src kinase, PLCγ, and the p85 subunit of PI 3-kinase. Recruitment of Src kinase is one of the first events associated with activation of FAK. Src kinase-induced transphosphorylation of Tyr576 and Tyr577 in the catalytic domain of FAK promotes maximal activation of FAK. Recruitment of FAK (or a FAK/Src kinase complex) to focal adhesions is facilitated by binding of membrane-associated p190 RhoGEF to the C-terminal targeting domain of FAK [16, 23].

The adaptor protein, paxillin, is a target for phosphorylation by FAK. Paxillin is bound in the cytosol to the scaffolding protein, vinculin, and mediates the recruitment of the paxillin-vinculin complex to focal adhesions in response to contractile stimulation [45–47]. Paxillin binds directly to FAK, and the binding of paxillin to FAK is necessary for the regulation of paxillin tyrosine phosphorylation [46–48]. ACh-induced paxillin phosphorylation at Tyr (Y118) was attenuated in cells expressing RhoA dominant negative (RhoA [T19N]) and by FAK inhibitor PF573228, but not by the Rho kinase inhibitor Y27632 in gastric smooth muscle cells. These results suggest that paxillin phosphorylation is downstream of RhoA and mediated by FAK but not Rho kinase. Paxillin associates with α-Pix, β-Pix and DOCK 180 GEF signaling molecules, which can regulate Cdc42 activity. Conversely, ACh-induced increase in the association of paxillin with α-Pix, β-Pix and DOCK 180 GEF signaling molecules and activation of Cdc42 was abolished in cells expressing RhoA dominant negative (RhoA [T19N]) indicating that activation of Cdc42 occurs via RhoA.

Activated Cdc42 binds directly to the CRIB (Cdc42 and Rac-interactive binding) domain of the nucleation promoting factor, N-WASp (neuronal Wiskott-Aldrich syndrome protein) [19, 29–32]. Actin polymerization by a contractile agonist is mediated by the N-WASp in airway and vascular smooth muscle [49, 28]. Activation of N-WASp undergoes a rearrangement that enables it to bind to the Arp complex. The Arp2/3 complex creates a template for actin polymerization that facilitates the addition of monomeric G -actin to existing F-actin filaments [32, 50, 51]. Thus, the activation of N-WASp is directly and specifically regulated by the binding of the small GTPase Cdc42 to its CRIB domain [29–32, 50]. Neither Rac nor Rho GTPase can bind directly to WASP family proteins; thus, RhoA cannot directly regulate N-WASp activity [29, 34].

To determine whether RhoA and Cdc42 activation are upstream regulators of N-WASp activation in gastric smooth muscle cells, we evaluated their role in the phosphorylation of N-WASP, the association of N-WASP with the Arp2/3 complex, and actin polymerization. RhoA and Cdc42 inactivation was found to inhibit N-WASP activation and its association with the Arp2/3 complex. We conclude that the activation of N-WASP and its association with the Arp2/3 complex are mediated by the activation of Cdc42, which is downstream of RhoA activation.

The inactivation of RhoA and Cdc42 was also found to inhibit the ACh induced increase in F/G-actin ratio (i.e., actin polymerization). ACh-induced increase in actin polymerization was also inhibited by the FAK inhibitor PF573228 and Arp2/3 complex inhibitor CK 666, but not by the Rho kinase inhibitor Y27632 indicating that actin polymerization is downstream of RhoA and Cdc42 activation. In this respect, the signaling mechanism of actin polymerization is similar to the airway smooth muscle. Further, the ACh-induced increase in sustained muscle contraction was abolished by C3 exoenzyme, Rho kinase inhibitor, FAK inhibitor, cytochalasin D, latrinculin, and Arp2/3 inhibitors but not by MLCK inhibitor ML-9. The effectiveness of the inhibitors such as Y27632, PF573228, cytochalsin D, latruculin and CK666 to block contraction in muscle strips in response to acetylcholine, the main excitatory neurotransmitter, suggests the role of actin polymerization in regulation of muscle contraction.

Our previous studies have shown that activation of muscarinic M3 receptors phosphorylates MYPT1 by Rho kinase to cause inhibition of MLC phosphatase and resulted in sustained MLC_20_ phosphorylation and contraction. We postulated that during the initial phase, Ca^2+^, not RhoA, would be the trigger for distinct pathways: one involving MLCK-induced MLC_20_ phosphorylation as previously reported [1, 3, 4], and the other involving Ca^2+^ dependent activation of Pyk2 and downstream effectors that mediate actin polymerization. Recent studies have shown that KCl-induced Ca^2+^ entry in smooth muscle stimulates Pyk2 activity in vascular smooth muscle (22). In our studies, IP_3_-induced Ca^2+^ release during the initial phase activated Pyk2 and stimulated Pyk2 phosphorylation of paxillin at Tyr118, the same Tyr residues phosphorylated by the homologous tyrosine kinase, FAK [47]. The phosphorylation of paxillin at these sites facilitates the association of paxillin with Cdc42 GEFs, and induces the sequential activation of Cdc42, N-WASP, and Arp2/3, resulting in actin polymerization and initial smooth muscle contraction. These results suggest that initial actin polymerization is Ca^2+^ dependent pathway via Pyk2. Xie et al showed lack of Pyk2 phosphorylation in mouse fundus in response to electrical field stimulation 5 s only [52]. In our study, when dispersed muscle cells were treated with acetylcholine for different time points starting from 30s to 5 min, minimal, but significant, Pyk2 phosphorylation was obtained at 30s and maximum response was obtained at 5 min. Thus, the discrepancy in data with Pyk2 phosphorylation could be due to experimental conditions.

One limitation of the current study is the incomplete time course of FAK and PYK2 phosphorylation. Previous research indicates that FAK (Y397) phosphorylation was active up to 70 min in N18TG2 neuroblastoma and phosphorylation of Pyk2 (Y402) was inhibited after 30 min and abolished by 180 min in rat aortic smooth muscle cells [53, 54]. However, it has not been evaluated in gastrointestinal smooth muscle. Therefore, a potential follow up study would examine FAK and PYK2 phosphorylation using an extended time course in our model. In addition, the present study did not examine tetrodotoxin (TTX) in muscle strips to evaluate neural activity. While there is possibility that neurons could be involved in the muscle strip contraction results presented here, the majority of the studies used smooth muscle cells, indicating that any potential neuronal activity does not play a major role.

While vascular smooth muscle contraction is similar to gastrointestinal smooth muscle contraction, in that actin polymerization requires FAK, PYK2, and Paxillin signaling pathways, vascular smooth muscle additionally activates the Src and CAS pathways, which have not been examined in gastrointestinal smooth muscle actin polymerization. For example, increased force generation by actin polymerization is activated by PKC mediated phosphorylation of paxillin, cofilin, and HSP27 and Rho kinase mediated phosphorylation of cofilin and HSP27 in rat cerebral artery [55, 56]. Furthermore, actin polymerization and blood pressure regulation in mouse arterial smooth muscle is mediated by the expression of vinculin and paxillin, which modulates p130 Crk associated substrate (CAS) activation through the non-receptor tyrosine kinase Abelson tyrosine kinase [57]. Therefore, a future direction may be to examine the importance of Src, CAS, CrkII, and vinculin pathway.

In summary, our studies suggest a novel mechanism for the regulation of smooth muscle contraction by Ca^2+^ dependent and Ca^2+^ independent pathways via actin polymerization. In gastric smooth muscle cells, IP_3_-induced Ca^2+^ release and activation of RhoA by the muscarinic M3 receptor regulates Pyk2, FAK, and paxillin. IP_3_- induced Ca^2+^ release during the initial phase activates Pyk2 and stimulates Pyk2 phosphorylation of paxillin at Tyr^118^. For the sustained phase, FAK binds to paxillin and phosphorylates it at Tyr^118^ by Ca^2+^ independent activation of RhoA. Phosphorylated paxillin associates with α-pix, β-pix and DOCK 180 signaling molecules. These GEF proteins commit to the activation of Cdc42 leading to the activation of N-WASP, the association of N-WASP with Arp2/3, actin polymerization, and muscle contraction that is independent of MLC_20_ phosphorylation. Our studies suggest a novel signaling pathway for gastric smooth muscle contraction via Ca^2+^ dependent phosphorylation of Pyk2 and Ca^2+^ independent phosphorylation of FAK. In this way, the phosphorylation of Pyk2, FAK, and paxillin plus the activation of downstream effectors, mediate actin polymerization in gastric smooth muscle (Fig 16).

**Fig 16:** Pathways mediating initial and sustained contraction via actin polymerization by ACh. Initial contraction and actin polymerization induced by acetylcholine involve G_q_-dependent PLC- activation, IP_3_ generation and Ca^2+^ release, and Ca^2+^ dependent activation of Pyk2. Sustained contraction and actin polymerization involve G_12/13_-dependent activation of RhoA, which recruits focal adhesion proteins such as FAK and paxillin to the membrane. FAK and paxillin interact at the adhesome. Phosphorylation of paxillin by activated FAK and Pyk2 facilitates the formation of complex containing paxillin with the Cdc42 GEFs, Pix and DOCK 180. This complex induces activation of Cdc42. Activation of Cdc42 in turn catalyzes the activation of neuronal Wiskott-Aldrich syndrome protein (N-WASp), which interacts with Arp2/3 complex to induce actin polymerization and muscle contraction.
